# Exosomal miR-221-3p Derived from Bone Marrow Mesenchymal Stem Cells Alleviates Asthma Progression by Targeting FGF2 and Inhibiting the ERK1/2 Signaling Pathway

**DOI:** 10.1155/2022/5910874

**Published:** 2022-08-10

**Authors:** Weike Liu, Hui Lin, Wuhui Nie, Jieting Wan, Qian Jiang, Aimei Zhang

**Affiliations:** ^1^Department of Pediatrics, Chengyang District People's Hospital of Qingdao, Qingdao 266000, Shandong, China; ^2^Department of Haemodialysis, Jimo District People's Hospital of Qingdao, Qingdao 266000, Shandong, China

## Abstract

Exosomes derived from human bone marrow mesenchymal stem cells (BMSCs) play potential protective roles in asthma. However, the underlying mechanisms remain not fully elucidated. Herein, exosomes were isolated from BMSCs, and the morphology, particle size, and exosome marker proteins were identified by transmission electron microscopy (TEM), nanoparticle tracking analysis (NTA), and Western blot, respectively. Then airway smooth muscle cells (ASMCs) were treated with transforming growth factor-*β*1 (TGF-*β*1) to construct a proliferation model and then incubated with BMSCs-derived exosomes. We found that exosome incubation increased miR-221-3p expression and inhibited proliferation, migration, and the levels of extracellular matrix (ECM) proteins including fibronectin and collagen III. Moreover, FGF2 was identified as a target gene of miR-221-3p. FGF2 overexpression reversed the inhibitory effects of exosomal miR-221-3p on ASMC progression. Besides, the phosphorylation of extracellular signal-regulated kinase 1/2 (ERK1/2) is inhibited by exosomal miR-221-3p, which was reversed by FGF2 overexpression. And ERK1/2 signaling activator reversed the effects of exosomal miR-221-3p on ASMC progression. Additionally, an ovalbumin (OVA)-induced asthmatic mice model was established, and exosome treatment alleviated airway hyper-responsiveness (AHR), histopathological damage, and ECM deposition in asthmatic mice. Taken together, our findings indicated that exosomal miR-221-3p derived from BMSCs inhibited FGF2 expression and the ERK1/2 signaling, thus attenuating proliferation, migration, and ECM deposition in ASMCs and alleviating asthma progression in OVA-induced asthmatic mice. Our findings may provide a novel therapeutic strategy for asthma.

## 1. Introduction

Asthma is a common chronic respiratory disease with high morbidity and mortality among children worldwide [1]. It is a complex syndrome characterized by airway hyper-responsiveness (AHR), airway inflammation, and airway remodeling [2]. Airway remodeling is involved in asthma progression through multifaceted processes including basement membrane thickening, extracellular matrix (ECM) deposition and abnormal airway smooth muscle cell (ASMC) growth [3, 4]. It has been emphasized that the abnormal proliferation and migration of AMSCs leads to airway wall thickening and airway narrowing and obstruction, which contributes to airway remodeling and severely affects lung function in patients with asthma [5]. Transforming growth factor-*β*1 (TGF-*β*1) was found to be elevated in the airway of patients with asthma, which facilitated airway remodeling by inducing ECM protein production and promoting ASMC proliferation and migration [6]. Although asthma symptoms can be relieved in children with asthma through several therapeutic methods, there is no available complete cure for childhood asthma up to now. Thus, novel effective therapeutic strategies based on a better understanding of molecular mechanisms of childhood asthma progression are urgently needed.

Bone marrow mesenchymal stem cells (BMSCs) are self-replicating multipotent stromal cells extracted from bone marrow mesenchymal tissues. Recently, accumulating evidence showed that BMSCs played a critical role in the treatment of autoimmune diseases including asthma due to their potent anti-inflammatory and immunomodulatory properties [7]. Importantly, it was found that the therapeutic function of BMSCs mainly depended on cell-to-cell communication through the secretion and transfer of exosomes [8]. Exosomes are small enclosed vesicles with a diameter of 50 to 150 nm, which are secreted by various types of cells and engaged in intercellular communication through transportation of functional signaling factors such as proteins, lipids, mRNAs, and microRNAs (miRNAs) [9]. The regulative role of BMSCs-derived exosomes in asthma has been identified in several types of research. For instance, BMSCs-derived exosomes promoted immunosuppression of regulatory T cells in asthma, indicating the therapeutic potential of BMSCs-derived exosomes for asthma [10]. BMSCs-derived exosomes inhibited airway remodeling and epithelial-mesenchymal transition of the airway epithelium in the lungs of asthmatic rats [11]. However, the regulatory mechanisms of BMSCs-derived exosomes in asthma progression have not been explored clearly.

MiRNAs are a class of small non-coding RNAs that regulate the post-transcriptional expression of target genes to mediate multiple biological and pathological processes. Increasing studies have demonstrated that exosomal miRNAs derived from BMSCs are involved in asthma development. A study suggested that there were different miRNA and mRNA profiles after BMSCs treatment in an asthma mouse model, and the miR-21/activin A receptor IIA axis is an important mechanism for the induction of asthmatic inflammation [12]. Moreover, BMSCs exosomal miR-1470 exerted an immunomodulatory effect by promoting the differentiation of CD4^+^CD25^+^FOXP^3+^ Tregs in asthmatic patients [13]. Interestingly, it was found that epithelial, sputum, and plasma miR-221-3p expression was significantly decreased in patients with asthma. The decreased expression of miR-221-3p might protect against airway eosinophilic inflammation by upregulating anti-inflammatory chemokine (C-X-C motif) ligand (CXCL) 17 (CXCL17) [14]. Likewise, miR-221-3p was found to have existed in the BMSCs-derived exosomes, and miR-221-3p delivered by BMSCs-derived exosomes was found to be involved in human physiological diseases such as acute myelocytic leukemia and ischemic stroke [15, 16]. Thus, we explored the roles of exosomal miR-221-3p derived from BMSCs in asthma progression.

In the present study, we investigated the effects and regulatory mechanism of exosomal miR-221-3p derived from BMSCs on TGF-*β*1-induced proliferation, migration, and ECM deposition in ASMCs, and then verified its effect on asthma progression in ovalbumin (OVA)-induced asthmatic mice, aiming to provide a novel therapeutic target for asthma.

## 2. Materials and Methods

### 2.1. BMSC Isolation and Culture

The Sprague-Dawley (SD) rats aged 6 weeks old were supplied by the Laboratory Animal Center of Shandong University. BMSCs were isolated according to the previously reported method [17]. The rats were euthanized through intraperitoneally anesthetizing with 1% pentobarbital sodium (100 mg/kg), and bone marrow was obtained from the femur and tibia of each rat under aseptic conditions. The bone marrow was centrifuged at 1000 g for 5 min, and the BMSCs precipitation was collected and suspended with Dulbecco's Modified Eagle Medium (DEME, Gibco, Grand Island, NY) supplemented with 10% fetal bovine serum (FBS; Gibco, Grand Island, NY), 100 U/mL penicillin and 100 *μ*g/mL streptomycin (Invitrogen, Carlsbad, CA, USA). BMSCs were cultured under humidified conditions with 5% CO_2_ at 37°C. The medium was changed in half volume after incubation for 24 h and then the whole medium was changed every 2 days. Cells were passaged at a confluence level of 80–90% at a ratio of 1 : 2.

### 2.2. Extraction and Identification of Exosomes from BMSCs

BMSCs in passage 3 with 80% confluence were selected for exosome extraction. BMSCs-derived exosomes were extracted by ultra-highspeed centrifugation [18]. In brief, the culture medium of BMSCs was successfully centrifuged at 300*g* for 10 min, 2000*g* for 10 min, and 10,000*g* for 35 min, and the supernatant was collected each time. Then the supernatant was filtered by using a 0.22 *μ*m filter membrane (Merck Millipore, Tullagreen, Ireland), followed by ultracentrifugation and centrifugation both 100,000*g* for 2 h, respectively. Finally, the exacted exosomes were collected, resuspended in phosphate-buffered saline (PBS), and stored at −80°C. The protein quality of exosomes was determined by the BCA Protein Assay Kit (Takara Biotechnology, Dalian, China). The levels of exosomal surface marker proteins including CD9, CD63, CD81, and TSG101 were detected by Western blot assay. The exosome morphology was identified by using Transmission electron microscopy (TEM, Hitachi, Tokyo, Japan), and the particle size of the extracted exosomes was measured by nanoparticle tracking analysis (NTA; Malvern Panalytical, Malvern, UK).

### 2.3. ASMC Culture and Treatment

ASMCs were obtained from patients without asthma who underwent lung resection surgery (*N* = 6) at the Chengyang District People's hospital of Qingdao City. Informed consent was obtained from each patient, and this study was approved by the Ethics Committee of Chengyang District People's hospital of Qingdao City. ASMCs were obtained according to a reported method [19]. In brief, the smooth muscle layer was isolated from healthy segments of the lobar or main bronchus of subjects through dissecting microscope. The tissues were washed with ice-cold PBS solution containing penicillin-streptomycin three times, and then were cut into small pieces and digested in Hanks' balanced salt solution (HBSS) containing 0.1% collagenase solution (Sigma, St. Louis, MO, USA) at 37°C for 30 min. Then the isolated cells were collected by centrifugation and cultured in DEME supplemented with 10% FBS, 100 U/mL penicillin, and 100 *μ*g/mL streptomycin under humidified conditions with 5% CO_2_ at 37°C. Cells cultured from 3 to 5 passages were used for subsequent experiments. ASMCs were stimulated with TGF-*β*1 (10 ng/mL; *R* & *D* Systems, Minneapolis, MN, USA) for 24 h to induce the proliferation model, and 100 *μ*g/mL exosomes were used to incubate with ASMCs in each group.

### 2.4. Cell Transfection

MiR-221-3p mimic (5′‐AGC UAC AUU GUC UGC UGG GUU UC‐3′), miR-221-3p inhibitor (5′‐GAA ACC CAG ACA AUG UAG CU‐3′) and their corresponding negative controls (NC mimic, NC inhibitor), and overexpression plasmids of fibroblast growth factor 2 (FGF2) (pcDNA-FGF2) and its negative control (vector) were obtained from RiboBio (Guangzhou, China). AMSCs were seeded in 6-well plates at 37°C in 5% CO_2_. When the cells grew to 80% confluence, Lipofectamine 3000 Transfection Reagent (Invitrogen, Carlsbad, CA) was used to transfect NC mimic (50 nM), miR-100-5p mimic (50 nM), NC inhibitor (50 nM), miR-100-5p inhibitor (50 nM), vector (30 nM), and pcDNA-FGF2 (30 nM) into AMSCs according to the manufacturer's instructions. Cells were collected after transfection for 48 h for further experiments.

### 2.5. Real-Time Quantitative Polymerase Chain Reaction (RT-qPCR)

Total RNA was extracted from ASMCs or lung tissues by using the TRIzol reagent (Invitrogen, Carlsbad, CA) according to the manufacturer's instructions. The cDNA synthesis was performed by using a PrimeScript RT reagent Kit (Takara Biotechnology, Dalian, China). Real-time quantitative polymerase chain reaction (RT-qPCR) was conducted with the SYBR Premix Ex Taq II (Takara, Dalian, China) on an Applied Biosystems 7500 Real-time PCR System (Applied Biosystems; Thermo Fisher Scientific, Inc.) under the following conditions: 95°C for 1 min, followed by 35 cycles of 95°C for 20 s, then 56°C for 10 s and 72°C for 15 s. The relative expression of miR-221-3p and FGF2 was normalized with U6 and glyceraldehyde 3-phosphate dehydrogenase (GAPDH), respectively. The relative expression levels were calculated by 2^−ΔΔCT^ method. The primers used are as follows: miR-221-3p (forward 5′-GAA ATG ATT CCA GGT AGC-3′ and reverse 5′-TGA ACA TCC AGG TCT GGG GCA-3′); U6 (forward, 5′-TGC GGG TGC TCG CTT CGG CAG C-3′, reverse, 5′-CCA GTG CAG GGT CCG AGG T-3′); FGF2 (forward, 5′-GCG ACC CAC ACG TCA AAC TA-3' and reverse, 5′-CTT AGA AGC CAG CAG CCG T-3′), GAPDH (forward: 5′-GGC AAA TTC AAC GGC ACA GT-3′, and reverse: 5′- GGC CTC ACC CCA TTT GAT GT-3′).

### 2.6. Western Blot Analysis

Proteins were extracted from ASMCs or lung tissues by using RIPA lysis buffer (Beyotime, Shanghai, China), and quantified by using the BCA method (Millipore, Billerica, MA, USA). Then the equal amount of protein (20 *μ*g) was subjected to 10% sodium dodecyl sulfate-polyacrylamide gel electrophoresis (SDS-PAGE) under the following conditions: 70 V for 30 min, followed by 120 V for 90 min. And then the protein bands were transferred to polyvinylidene difluoride (PVDF) membranes (Millipore, Bedford, MA, USA) at 300 mA for 2 h. The membranes were blocked with 5% nonfat milk for 1 h at room temperature and then incubated overnight at 4°C with the following primary antibodies obtained from Abcam (Cambridge, UK): anti-CD63 antibody (1 : 1000, ab134045), anti-CD9 antibody (1 : 1000, ab236630), anti-CD81 antibody (1 : 1000, ab109201), anti-TSG101 antibody (1 : 1000, ab125011), anti-FGF2 antibody (1 : 1000, ab208687), anti-fibronectin antibody (1 : 1000, ab45688), anti-collagen III antibody (1 : 1000, ab184993), anti-ERK1/2 antibody (1 : 1000, ab17942), anti-ERK1/2 antibody (phospho T202 + Y204) (1 : 1000, ab214362), and anti-GAPDH antibody (1 : 2500, ab9485). Then the membranes were incubated with horseradish peroxidase (HRP)-conjugated goat anti-rabbit IgG (1 : 2000, Abcam, ab6721) for 1 h. The protein bands were visualized with ECL detection reagents and analyzed with ImageJ software (National Institutes of Health, Bethesda, MA, USA).

### 2.7. CCK-8 Assay

Cell proliferation was measured by using the Cell Counting Kit-8 (CCK-8, Dojindo, Japan) assay. Briefly, ASMCs were seeded into 96-well plates at a density of 1 × 10^4^ cells/well. After incubation for 0, 24, 48, and 72 h at 37°C, 10 *μ*L of CCK-8 solution was added to each well and incubated for 2 h at 37°C. The absorbance at 450 nm of each well was measured by using a microplate reader (Molecular Devices, Shanghai, China).

### 2.8. Transwell Migration Assay

A Transwell assay was performed to measure ASMC migration. Briefly, HTR8/SVneo cells with the serum-free medium were seeded into the upper chamber of Transwell chambers (8.0 *μ*m pore size; Millipore Corporation, USA). And the DMEM medium was added to the lower chamber. After culturing for 24 h at 37°C, cells on the upper chamber were removed by using a cotton swab, while the cells in the bottom chamber were fixed with 70% ethanol for 10 min and stained with 0.1% crystal violet for 15 min. The migrated cells were quantified by counting five random fields at ×200 magnification under a light microscope (Olympus, Tokyo, Japan).

### 2.9. Dual-Luciferase Reporter Gene Assay

The potential targets of miR-221-3p were predicted by using the online bioinformatics tool Starbase (https://starbase.sysu.edu.cn/). The binding sites at FGF2 3′-UTR were mutated from AUGUACC to CCCCGAA and then cloned into the pGL3-control luciferase reporter vectors (Promega, Madison, WI) to construct the wild-type (FGF2-WT) and mutant type (FGF2-MUT) reporter vector. Then the reporter plasmids and miR-221-3p mimic or NC-mimic were co-transfected into ASMCs. Following transfection for 48 h, relative luciferase activity was measured by using the Dual Luciferase Reporter Assay System (Promega, Madison, Wisconsin, WI, USA).

### 2.10. Animal Experimental Protocols

BALB/c mice (6–8 weeks old, 20 ± 2 g) were obtained from the Laboratory Animal Center of Shandong University, which were maintained in sterile cages under 22–25°C temperature, 55–60% humidity, and 12 h light/dark cycle conditions with free access to food and water. All animal experiments in this study were approved by the Animal Ethics Committee of Laboratory Animal Center of Shandong University.

Mice were randomly divided into three groups (*n* = 8 per group): control group, OVA group, and OVA + Exo group. The Asthma mouse model was established as previously described [20]. The mice in the OVA group were sensitized on days 0, 7, and 14 by intraperitoneal injection of 20 *μ*g of ovalbumin (OVA), emulsified in 1 mg aluminum hydroxide in a total volume of 200 *μ*L. Then the mice were exposed to a 1% OVA aerosol for up to 1 h From day 21 to 23. The mice in the control group were treated with an equal volume of saline instead of OVA. For exosome treatment, 100 *μ*g of exosomes in 100 *μ*L PBS was intratracheally administered every day on days 21 to 23. All mice were euthanized 24 h for the subsequent procedures after the last OVA challenge.

### 2.11. Measurement of Airway Hyperresponsiveness

Within 24 h after the last OVA challenge, mice were anesthetized with 1% pentobarbital sodium and subjected to mechanical ventilation, and the airway hyperresponsiveness (AHR) of mice was measured by using an animal pulmonary function instrument (Buxco, CT, USA). Subsequently, all mice were exposed to increasing doses of methacholine aerosol (Sigma-Aldrich, USA) at 0, 5, 10, 25, and 50 mg/mL for 3 min, and the enhanced pause (Penh) value of unrestrained mice within 5 min was recorded according to the protocols of the instrument.

### 2.12. Histopathological Evaluation

The rats were euthanized through intraperitoneally anesthetizing with 1% pentobarbital sodium (100 mg/kg). Lung tissues were collected, fixed with paraformaldehyde, and embedded with paraffin. Then the tissues were cut into 5 *μ*m thick sections and stained with hematoxylin and eosin (HE) using a standard protocol and analyzed by light microscopy (magnification ×200; Olympus, Tokyo, Japan).

Lung tissues were subjected to Masson trichrome staining to determine collagen deposition. Tissue sections were stained with hematoxylin solution for 6 min, ponceau and acid fuchsin solution for 1 min, and phosphomolybdic acid solution for 5 min. And then restained with aniline blue solution for 5 min. The tissue sections were analyzed by light microscopy (magnification ×400; Olympus, Tokyo, Japan).

### 2.13. BALF Collection and Cell Counting

After mice were anesthetized, the tracheas were cannulated and lavaged with 0.8 mL of cold PBS twice to collect bronchoalveolar lavage fluid (BALF). The BALF samples were immediately centrifuged at 300*g* for 15 min to collect the supernatant. The number of total cells in BALF was determined with a hemocytometer. The differences in cell number of eosinophils, neutrophils, lymphocytes, and macrophages in BALF were evaluated by using the Kwik-Diff staining set (Thermo, USA) according to the manufacturer's instructions.

### 2.14. Measurement of the Serum Level of OVA-Specific IgE

On day 24 after the last OVA challenge, the blood samples of mice were collected and centrifuged at 1000*g* for 10 min to obtain serum samples. The serum level of OVA-Specific immunoglobulin E (IgE) was measured by ELISA kit (Abcam, Cambridge, UK) according to the manufacturer's instructions.

### 2.15. Statistical Analysis

Statistical analysis was performed by using SPSS version 22.0 software. All data from at least three times independent experiments were presented as mean ± standard deviation (SD). Student's *t*-test and analysis of variance (ANOVA) followed by Tukey-Kramer correction were performed for the comparison between two groups and comparison among groups, respectively. *P* < 0.05 was considered to be statistically significant.

## 3. Results

### 3.1. Identification of Exosomes Isolated from BMSCs

We first identified the isolated exosomes from BMSCs. The expression of exosome-specific markers, including CD9, CD63, CD81, and TSG101 was measured by Western blotting, which showed that all exosome marker levels were significantly higher in the isolated exosomes than that in BMSCs and supernatant (Figures 1(a) and 1(b)). Moreover, the exosome morphology was identified by TEM (Figure 1(c)) and NTA revealed that the mean particle size of exosomes was 134.2 nm (Figure 1(d)). These results indicated that BMSCs-derived exosomes were successfully obtained in our experiments.

### 3.2. Exosomal miR-221-3p Derived from BMSCs Inhibited Proliferation, Migration, and ECM Deposition in ASMCs

To explore whether exosomal miR-221-3p derived from BMSCs is involved in childhood asthma progression, ASMCs were treated with TGF-*β*1 to induce a proliferation model and then incubated with BMSCs-derived exosomes alone or together with transfection with miR-221-3p inhibitor. RT-qPCR showed that the level of miR-221-3p was decreased in TGF-*β*1-treated ASMCs, and exosome incubation upregulated miR-221-3p level, while transfection of miR-221-3p inhibitor reduced miR-221-3p level (Figure 2(a)). Moreover, it was observed that TGF-*β*1 stimulation promoted cell proliferation (Figure 2(b)) and migration (Figures 2(c) and 2(d)) in ASMCs, and exosome incubation markedly attenuated proliferation and migration, while miR-221-3p inhibition reversed these effects. Additionally, ASMCs play an important role in airway remodeling by producing ECM proteins. We next determined the functional role of exosomal miR-221-3p in TGF-*β*1-induced ECM deposition. Western blotting demonstrated that TGF-*β*1 stimulation induced the expression of fibronectin and collagen III in ASMCs, and exosome incubation significantly decreased the expression of fibronectin and collagen III, which were then reversed by miR-221-3p inhibition (Figures 2(e)–2(g)). These results indicated that exosomal miR-221-3p derived from BMSCs inhibited proliferation, migration, and ECM deposition in ASMCs.

### 3.3. FGF2 is a Target Gene of miR-221-3p

The potential target mRNAs of miR-221-3p were predicted by using the StarBase tool (https://starbase.sysu.edu.cn/), which suggested that there were potential binding sites between miR-221-3p and FGF2 (Figure 3(a)). Dual luciferase reporter gene assay further confirmed that only the relative luciferase activity of FGF2-WT was significantly inhibited after transfection with miR-221-3p mimic, while the relative luciferase activity of FGF2-MUT was not affected by any treatment (Figure 3(b)). Furthermore, miR-221-3p mimic, miR-221-3p inhibitor, and their negative controls were transfected into ASMCs, respectively. As shown in Figure 3(c), the expression of miR-221-3p in ASMCs was increased in the miR-221-3p mimic group and decreased in the miR-221-3p inhibitor group. Moreover, miR-221-3p overexpression apparently inhibited the expression of FGF2 at both mRNA and protein levels, while miR-221-3p inhibition markedly promoted the mRNA and protein expression of FGF2 (Figures 3(d)–3(f)). These findings indicated that FGF2 was a target gene of miR-221-3p.

### 3.4. Exosomal miR-221-3p Inhibited Proliferation, Migration, and ECM Deposition in ASMCs by Downregulating FGF2

To further investigate whether miR-221-3p exerts its function by regulating FGF2 in ASMCs, TGF-*β*1-treated ASMCs were incubated with BMSCs-derived exosomes alone or together with transfection with pcDNA-FGF2. We found that TGF-*β*1 stimulation upregulated the mRNA and protein levels of FGF2 in ASMCs, and exosome incubation reduced the mRNA and protein levels of FGF2, whereas transfection of pcDNA-FGF2 promoted the mRNA and protein expression of FGF2 (Figures 4(a)–4(c)). Moreover, CCK-8 and Transwell assays illustrated that exosome incubation inhibited TGF-*β*1-induced proliferation (Figure 4(d)) and migration (Figures 4(e) and 4(f)) in ASMCs, while FGF2 overexpression reversed these effects. Additionally, Western blotting showed that exosome incubation significantly decreased TGF-*β*1-induced fibronectin and collagen III production in ASMCs, which were abolished by FGF2 overexpression (Figures 4(b), 4(g), and 4(h)). These results implicated that exosomal miR-221-3p inhibited proliferation, migration, and ECM deposition in ASMCs by downregulating FGF2.

### 3.5. The ERK1/2 Signaling is Involved in the Regulation of Exosomal miR-221-3p/FGF2 Axis on ASMC Progression

We further explored whether the extracellular regulated protein kinases 1/2 (ERK1/2) signaling is perturbed by the exosomal miR-221-3p/FGF2 axis in ASMCs. Western blotting revealed that exosomal miR-221-3p incubation significantly decreased TGF-*β*1-induced phosphorylated ERK1/2 (p-ERK1/2) expression in ASMCs, while FGF2 overexpression increased p-ERK1/2 expression (Figures 5(a) and 5(b)). To confirm whether the ERK1/2 signaling is involved in the regulation of exosomal miR-221-3p/FGF2 axis on ASMC progression, TGF-*β*1-treated ASMCs were incubated with BMSCs-derived exosomes in the absence or presence of ERK1/2 signaling activator tert-butylhydroquinone (TBHQ). It was found that exosomal miR-221-3p incubation suppressed p-ERK1/2 expression in ASMCs, while TBHQ treatment enhanced p-ERK1/2 expression (Figures 5(c) and 5(d)). Furthermore, exosomal miR-221-3p incubation attenuated TGF-*β*1-induced proliferation (Figure 5(e)), migration (Figures 5(f) and 5(g)) and ECM protein production (Figures 5(h)–5(j)) in ASMCs, while TBHQ treatment reversed these effects. These results revealed that the exosomal miR-221-3p/FGF2 axis modulated ASMC progression by regulating the ERK1/2 signaling.

### 3.6. Exosomal miR-221-3p Derived from BMSCs Alleviated Asthma Progression in Mice

To further explore the role of exosomal miR-221-3p in asthma progression *in vivo*, the OVA-induced asthmatic mice model was constructed, and exosomal miR-221-3p was injected for treatment. We confirmed the decreased miR-221-3p expression (Figure 6(a)) and increased FGF2 expression (Figures 6(b) and 6(c)) in lung tissues of the OVA group compared with the control group, and this expression pattern was reversed by exosomal miR-221-3p treatment. Then the airway hyperresponsiveness was detected by measuring the Penh value, which showed that aerosolized methacholine caused a dose-dependent increase in Penh value in all groups, and the Penh value in the OVA group was higher than that in the control group, while exosomal miR-221-3p treatment significantly reduced the Penh value in OVA-challenged mice (Figure 6(d)). Next, histopathological evaluation of lung tissue sections from each group was detected by HE staining and Masson staining. HE staining showed that OVA-challenged mice showed obvious inflammatory cell infiltration and bronchial wall thickening, while exosomal miR-221-3p treatment attenuated these histopathological changes (Figure 6(e)). Masson staining indicated that a large amount of collagen deposition around the bronchioles in the OVA group, while exosomal miR-221-3p exerted a substantial effect on reducing ECM deposition (Figure 6(f)). Additionally, the number of inflammatory cells including neutrophils, eosinophils, macrophages, and lymphocytes in BALF was increased significantly in the OVA group compared with that in the control group, while treatment of exosomal miR-221-3p reduced the number of inflammatory cells (Figure 6(g)). ELISA results showed that the levels of serum OVA-specific IgE (Figure 6(h)) and inflammatory cytokines including TGF-*β*1, IL-3, and IL-14 levels (Figure 6(i)) were significantly elevated in lung tissues of OVA-challenged mice, while exosomal miR-221-3p treatment significantly reversed this effect. Our results revealed that exosomal miR-221-3p derived from BMSCs alleviated asthma progression in mice.

## 4. Discussion

Emerging evidence has revealed the potential protective role of BMSCs-derived exosomes in asthma progression due to their anti-inflammatory and immunomodulatory properties [7]. However, the possible underlying mechanisms of BMSCs-derived exosomes in the protection of asthma remain not fully understood. A large number of studies have confirmed that BMSCs-derived exosomes play crucial roles in the human pathological process through the transportation of functional miRNAs [7, 21]. A previous study illustrated that miR-221-3p delivered by BMSCs-derived exosomes promoted the development of acute myelocytic leukemia [15]. Moreover, BMSCs-derived extracellular vesicles carrying miR-221-3p exerted a neuroprotective effect in ischemic stroke by targeting activating transcription factor 3 [16]. Interestingly, it was found that epithelial, sputum and plasma miR-221-3p expression was prominently decreased in patients with asthma, and the decreased expression of miR-221-3p might protect against airway eosinophilic inflammation by upregulating anti-inflammatory chemokine CXCL17, indicating that epithelial and sputum miR-221-3p are novel biomarkers for airway eosinophilic inflammation in asthma [14]. Thus, our study investigated the roles and underlying mechanism of exosomal miR-221-3p derived from BMSCs in asthma progression. We found that exosomal miR-221-3p derived from BMSCs inhibited TGF-*β*1-induced proliferation and migration, and reduced the levels of ECM proteins including fibronectin and collagen III in ASMCs. Additionally, exosomal miR-221-3p alleviated AHR, histopathological damage, and collagen deposition in OVA-induced asthmatic mice. Importantly, we suggested that exosomal miR-221-3p achieved its protective roles by targeting fibroblast growth factor 2 (FGF2) in ASMCs.

FGF2, also known as the basic fibroblast growth factor (bFGF), is a potent mitogenic factor belonging to the FGF family. It was reported that FGF2 was overexpressed in asthma and promoted airway inflammation in airway epithelial cells [22]. Recently, studies have focused on the immunomodulatory function of FGF2 in chronic inflammatory airway diseases including asthma and chronic obstructive pulmonary disease [23]. Notably, FGF2 inhibited TGF-*β*1-induced differentiation of ASMCs in vitro [24]. Moreover, FGF2 and TGF-*β*1 synergized in human bronchial smooth muscle cell (BSMC) proliferation, and this synergistic effect might contribute to the hyperplastic phenotype of BSMC in asthmatic airway remodeling [25]. These studies indicated that FGF2 was involved in asthma progression and might be a therapeutic target for asthma diseases. In our study, we showed that FGF2 was a target gene of miR-221-3p, and FGF2 expression was inhibited by miR-221-3p in ASMCs, Furthermore, FGF2 overexpression reversed the inhibitory effect of exosomal miR-221-3p on TGF-*β*1-induced proliferation, migration, and ECM deposition in ASMCs, indicating that exosomal miR-221-3p exerted its protective role in asthma by inhibiting FGF2 expression.

The ERK1/2 signaling pathway is a common pathway regulated by various proliferative factors, which is identified as a pivotal factor in asthma progression [26]. And the role of ERK1/2 signaling in promoting the proliferation and migration of ASMCs was previously reported. Biased Bitter taste receptor (TAS2R) bronchodilators inhibited ASMC proliferation by downregulating phosphorylated ERK1/2 [27]. Vasoactive intestinal peptides inhibited airway remodeling in asthmatic mice, and inhibited phosphorylation of the ERK1/2 signaling on ASMCs, thus inhibiting the proliferation of ASMCs [26]. More notably, FGF2 is closely related to wound repair and cell proliferation. Recent studies provided us the evidence that FGF2 participated in regulating the ERK1/2 signaling in cell proliferation. For instance, FGF2 significantly enhanced liver cell proliferation by increasing the phosphorylation level of ERK1/2 and c-Jun N-terminal kinase (JNK) [28]. FGF2 promoted proliferation and migration of uterine luminal epithelial cells during early pregnancy, which was reversed by the treatment of inhibitor U0126 [29]. Therefore, we explored whether the ERK1/2 signaling is involved in the regulation of the miR-221-3p/FGF2 axis in ASMC progression. Our results illustrated that exosomal miR-221-3p suppressed FGF2-mediated phosphorylation of the ERK1/2 signaling, and ERK1/2 activator TBHQ reversed the inhibitory effects of exosomal miR-221-3p on proliferation, migration, and ECM deposition in ASMCs, indicating that exosomal miR-221-3p attenuated ASMC progression through inhibiting the ERK1/2 signaling [30].

In conclusion, our findings demonstrated that exosomal miR-221-3p derived from BMSCs inhibited FGF2 expression and the ERK1/2 signaling, thus attenuating proliferation, migration, and ECM deposition in ASMCs. Additionally, exosomal miR-221-3p alleviated asthma progression in OVA-induced asthmatic mice. Our findings may provide a novel therapeutic strategy for asthma.

## Figures and Tables

**Figure 1:** Identification of exosomes isolated from BMSCs. (a)-(b) The levels of exosome-specific markers, including CD9, CD63, CD81, and TSG101 in BMSCs, supernatant, and exosomes were measured by western blot analysis. ^*∗*^*P* < 0.05. (c) The exosome morphology was determined by transmission electron microscopy (TEM) (scale bar: 100 nm). (d) The particle size of exosomes was detected by nanoparticle tracking analysis (NTA). Data from at least three independent experiments were presented as mean ± SD ^*∗*^*P* < 0.05.

**Figure 2:** Exosomal miR-221-3p inhibited proliferation, migration, and ECM deposition in ASMCs. ASMCs were treated with TGF-*β*1 to induce a proliferation model and then incubated with BMSCs-derived exosomes alone or together with transfection with miR-221-3p inhibitor. (a) RT-qPCR was performed to measure the expression of miR-221-3p. (b) ASMC proliferation was evaluated by using the CCK-8 assay. (c), (d) ASMC migration was measured by using Transwell assay. (e)–(g) The protein expression of fibronectin and collagen III was analyzed by using western blot analysis. Data from at least three independent experiments were presented as mean ± SD ^*∗*^*P* < 0.05.

**Figure 3:** FGF2 is a target gene of miR-221-3p. (a) The binding sites of miR-221-3p were predicted by the starbase tool. (b) Dual-luciferase reporter gene assay verified the binding between miR-221-3p and FGF2. (c) ASMCs were transfected with miR-221-3p mimic, miR-221-3p inhibitor, and their negative controls, respectively. The expression of miR-221-3p was detected by RT-qPCR. (d) The expression of FGF2 mRNA was detected by RT-qPCR (e), (f) The expression of FGF2 protein was measured by using western blot analysis. Data from at least three independent experiments were presented as mean ± SD ^*∗*^*P* < 0.05.

**Figure 4:** Exosomal miR-221-3p inhibited proliferation, migration, and ECM deposition in ASMCs by downregulating FGF2. TGF-*β*1-treated ASMCs were incubated with BMSCs-derived exosomes alone or together with transfection with pcDNA-FGF2. (a) The expression of FGF2 mRNA was detected by RT-qPCR. (b), (c) The protein expression of FGF2 was detected by western blot analysis. (d) CCK-8 assay was performed to evaluate ASMC proliferation. (e), (f) Transwell assay was performed to detect ASMC migration. (g)-(h) The protein expression of fibronectin and collagen III was analyzed by using Western blot analysis. Data from at least three independent experiments were presented as mean ± SD ^*∗*^*P* < 0.05.

**Figure 5:** The ERK1/2 signaling is involved in the regulation of the exosomal miR-221-3p/FGF2 axis on ASMC progression. (a), (b) TGF-*β*1-treated ASMCs were incubated with BMSCs-derived exosomes alone or together with transfection with pcDNA-FGF2. The protein levels of p-ERK1/2 and ERK1/2 were detected by western blot analysis. TGF-*β*1-treated ASMCs were incubated with BMSCs-derived exosomes in the absence or presence of ERK1/2 signaling activator TBHQ. (c), (d) The protein levels of p-ERK1/2 and ERK1/2 were detected by western blot analysis. (e) ASMC proliferation was measured by using the CCK-8 assay. (f), (g) ASMC migration was measured by transwell assay. (h)–(j) The protein expression of fibronectin and collagen III was analyzed by using Western blot analysis. Data from at least three independent experiments were presented as mean ± SD ^*∗*^*P* < 0.05.

**Figure 6:** The exosomal miR-221-3p derived from BMSCs alleviated asthma progression in mice. BALB/c mice were randomly divided into three groups (*n* = 8 per group): control group, OVA group, and OVA + Exo group. OVA-induced asthmatic mice model was constructed, and exosomal miR-221-3p was injected for treatment. (a) The expression of miR-221-3p in lung tissues of mice was measured by using RT-qPCR. (b), (c) The expression of FGF2 protein in lung tissues of mice was detected by using Western blot analysis. (d) The airway hyperresponsiveness of mice in all groups was detected. (e), (f) Histopathological evaluation of lung tissue sections from each group were detected by HE staining and Masson staining, and significant histopathological changes were marked with an arrow. (g) The number of total and differential inflammatory cells in BALF. (h) The serum OVA-specific IgE levels of mice in all groups were detected by using ELISA.(i) The levels of TGF-*β*1, IL-4, and IL-13 in BALF were examined by using ELISA. Data from at least three independent experiments were presented as mean ± SD ^*∗*^*P* < 0.05.

## Data Availability

The datasets used during the present study are available from the corresponding author upon reasonable request.
